# Effects of Pamidronate Disodium Combined with Calcium on BMD Values and Severity of Pain in Elderly Patients with Osteoporosis Based on Mobile Terminal Platform for Internet of Things

**DOI:** 10.1155/2022/5069918

**Published:** 2022-08-16

**Authors:** Zuoming Bai, Jianguo Wang, Mingming Kang, Peng Guo, Dong Wang

**Affiliations:** Department of Orthopedics, The Second Hospital of Shanxi Medical University, Taiyuan, 030001 Shanxi, China

## Abstract

**Objective:**

To explore the effects of pamidronate disodium combined with calcium on BMD values and the severity of pain in elderly patients with osteoporosis based on the mobile terminal platform for the Internet of Things.

**Methods:**

The data of 120 patients admitted to our hospital from January 2019 to December 2020 were retrospectively analyzed. According to the patients' condition and medication wills, they were divided into the experimental group (*n* = 68) and the control group (*n* = 52). All patients were given chronic disease management based on the mobile terminals for the Internet of Things, and they received the treatment of bisphosphonates and calcium, with the supplement of calcium at a daily dose of 1000 mg. The control group was given alendronate sodium once a week, and the experimental group was given pamidronate disodium by intravenous infusion three times a month, with the treatment cycle as 1 year. The patients' bone mineral density (BMD) values and the pain indexes were compared after treatment.

**Results:**

There was no statistical difference in general information between the two groups (*p* > 0.05). The BMD values of the lumbar vertebrae L_2-4_, total hip, and femur neck at 6 months and 1 year after treatment in the experimental group were significantly higher than those in the control group (*p* < 0.001). The pain scores at 6 months and 1 year after treatment in the experimental group were significantly lower than those in the control group (*p* < 0.001).

**Conclusion:**

The treatment of pamidronate disodium combined with calcium based on the mobile terminal platform for the Internet of Things can reduce the severity of pain in elderly patients with osteoporosis and improve the BMD, which has a generalization value.

## 1. Introduction

Osteoporosis is a chronic progressive systemic metabolic osteopathy characterized by a low bone mineral density (BMD). The bone microarchitecture of patients is damaged, and the bone fragility is aggravated. Patients with mild conditions in the early stage have no obvious symptom, and the diffuse pain or even systemic osteodynia can occur with the progress of disease. The incidence of fractures significantly increases [1, 2], which seriously affects the patients' quality of life. In recent years, with the aggravation of the population aging in China, the incidence of osteoporosis has increased, and the relevant data predict that the number of patients with osteoporotic fractures will reach 6 million by 2050 in China with the corresponding medical expenditure more than RMB 100 billion [3, 4]. Therefore, the deepening of clinical research on osteoporosis is beneficial for reducing the future medical burden in China and improving the prognosis of elderly patients with osteoporosis. At present, calcium is the main medicine for the treatment of osteoporosis, but the calcium treatment alone cannot exert an ideal prevention and control effect, and elderly patients with low calcium absorption rate in intestinal tract and 1*α*-hydrolase activity of kidney cannot benefit from it [5, 6]. In addition to calcium, bisphosphonates are also the first-line drug for the treatment of osteoporosis, which can inhibit the bone remodeling, increase the BMD, improve the bone microarchitecture of patients, and reduce the possibility of fracture [7]. Since the bisphosphonates are prone to induce the adverse reactions, there are a few studies on the application of bisphosphonates in elderly patients with osteoporosis. Filippo et al. have found that zoledronic acid is the most likely to induce the adverse reactions, followed by pamidronate disodium and alendronate sodium [8]. This study did not compare the medication safety, which was the limitation of this study, but the safety of pamidronate disodium has been confirmed in various diseases. Pamidronate disodium has the same efficacy and the incidence of adverse reactions in alleviating and delaying the occurrence time of skeletal-related events in non-small-cell lung cancer with bone metastasis, and the use of zoledronic acid after ineffective treatment of pamidronate disodium can delay the occurrence time of skeletal-related events. Pamidronate disodium, as a new generation of bisphosphonates, can effectively inhibit the activity of osteoclasts, hinder the bone resorption mediated by osteoclasts, repair the osteolytic lesions, and slow down the rate of organismal bone resorption, thus exerting an impact on preventing the osteoporosis [9]. Most importantly, pamidronate disodium is often used in the treatment of bone metastasis of advanced malignant tumors. The medicine can inhibit the synthesis of osteoclasts and the release of nociceptive transmitters such as prostaglandin and reduce the symptoms of osteodynia, which plays an important role in improving the patients' quality of life. Most elderly patients with chronic diseases have the problem of low medication compliance, and low medication compliance is an important factor affecting the treatment effect of patients. Most literature shows that the compliance of elderly patients gradually decreases after leaving hospital; so, it is crucial to improve the medication compliance of patients. The mobile terminal platform for the Internet of Things can exert a monitoring role through multimode diagnosis and treatment, provide strong external support, and maintain medication compliance in elderly patients with osteoporosis. At present, there is no clinical research on the combined application of disodium pamidronate and calcium in the treatment of elderly osteoporosis. Based on the mobile terminal platform for the Internet of Things, in this study, the supervision and management of medication for elder patients with osteoporosis were strengthened, and the actual effects of pamidronate disodium combined with calcium in the treatment of elderly osteoporosis were explored. The reports are as follows.

## 2. Materials and Methods

### 2.1. Research Design

This retrospective study was conducted in our hospital from January 2019 to December 2020 to explore the effects of pamidronate disodium combined with calcium on BMD values and the severity of pain in elderly patients with osteoporosis based on the mobile terminal platform for the Internet of Things. The blind level of this study was double-blind. The study subjects and researchers did not understand the grouping of this experiment, and the research designers were responsible for arranging and controlling the experiment.

### 2.2. Inclusion and Exclusion Criteria

Inclusion criteria were as follows: (1) patients were diagnosed with primary osteoporosis according to the biochemical examination of bone metabolism in accordance with the diagnostic criteria of osteoporosis recommended by the International Society of Clinical Densitometry (ISCD) [10] and American college of radiology [11]. (2) Patients had the clinical manifestations with spontaneous pain in the whole body, waist, thorax, and back. (3) The BMD in patients measured by dual-energy absorptiometry was lower than 2.5 standard deviations below the mean in healthy people of the same age and sex. (4) Patients had not taken any drugs affecting the bone metabolism in the last three months. (5) The age of patients was more than 70 years old. (6) All patients were treated in our hospital during the whole process with the complete clinical information. (7) Patients were cooperative to complete the follow-up.

Exclusion criteria were as follows: (1) patients with secondary osteoporosis due to the endocrine metabolism, alimentary deficiency, and rheumatism; (2) patients who had taken drugs that might affect the bone metabolism in the last three months; (3) patients with the history of malignant tumor and cardiovascular disease or patients with the diseases that could affect the bone metabolism; (4) patients with the irrational drug use that might have the undefined treatment effects; (5) patients with the incomplete clinical information; (6) patients without complete follow-up; and (7) patients with psychiatric disorders and who could not communicate with others.

### 2.3. Procedures

In this study, 120 patients were divided into the experimental group (*n* = 68) and the control group (*n* = 52) according to the patients' condition and medication wills. All patients were given the chronic disease management based on the mobile terminals for the Internet of Things, and they received the treatment of bisphosphonates and calcium. On the day when the patients agreed to participate in the study, the study group collected the data of sociodemography and clinical manifestations. After the patients began to receive the treatment, they were given the follow-up for 1 year to investigate the changes of BMD and the pain perception.

### 2.4. Moral Consideration

This study was in line with the principles of Declaration of Helsinki (2013) [12], and patients signed the informed consent.

### 2.5. Standards of Withdrawing from Experiment

In the following conditions, the study group judged that patients were inappropriate for continuing the experiment, and the case record forms of patients were retained, but the data analysis was not performed: (1) patients with exacerbation during the experiment, (2) patients with severe comorbidities or complications, and (3) patients who requested the withdrawal from the clinical trials.

### 2.6. Methods

All patients were given the chronic disease management based on the mobile terminals for the Internet of Things, and the project of healthcare cloud was constructed. The integrated management system of osteoporosis was consolidated into the cloud platform to build a remote monitoring platform for osteoporosis medication. Patients needed to register and report on the mobile terminal platform, and they were supervised and managed through the mobile terminal platform for the Internet of Things.

Control group was as follows: the control group was given the alendronate sodium (Beijing Wansheng Pharmaceutical Co., Ltd.; NMPA approval No. H20058996) once a week at a single dose of 70 mg with 300 ml of warm water on an empty stomach in the morning. Patients should keep standing or sitting within half an hour after taking the medicine and then take food. In addition, patients were given calcium (Huishi Pharmaceutical Co., Ltd.; NMPA approval No. H10950029) at a daily dose of 600 mg and 2 pellets of active vitamin D (Sinopharm Xingsha Pharmaceutical Co., Ltd.; NMPA approval No. H20173093).

The experimental group was as follows: The supplement of calcium and vitamin D in the experimental group was the same as those in the control group. In addition, the pamidronate disodium (Shenzhen Haiwang Pharmaceutical Co., Ltd.; NMPA approval No. H19980130) at a single dose of 30 mg diluted in 250 ml of 5% glucose once a day on 3 consecutive days was given by intravenous infusion three times a month.

### 2.7. Standards of Observation

1. General information: the general information of patients such as gender, age, body mass, BMI, the course of disease, the severity of osteoporosis, education level, income level, payment of medical expenses, and the place of residence in the two groups were recorded
2. BMD: the BMD values of patients were detected before treatment and at 6 months and 1 year after treatment using a dual energy X-ray absorptiometry (DTX-200; NMPA (I) 20113302208) by Osteometer MediTech, USA. Before the examination, the precision of instruments was calibrated by the model of lumbar vertebrae with the coefficient of variation (CV) as 0.40%. After the patients kept lying flat, the bone scan of lumbar vertebrae (L_2-4_) in supine position was performed, and the hip was scanned in knee flexion position of both lower extremities. The BMD values of lumbar vertebrae, total hip, and femur neck were recorded
3. Pain indexes: before treatment, and at 6 months and 1 year after treatment, the patients' severity of pain was evaluated with an 11-spot numeric rating scale (NRS). In the scale, the number of 0-10 on the straight line represented the severity of pain, and the patients chose the spot which was consistent with the severity of pain according to their own condition after visual estimation. 0 point represented the painlessness, 1-3 points represented the mild pain that did not interfere with sleep, 4-6 points represented the moderate pain, 7-9 points represented the severe pain that could not fall asleep or woke up from the pain during sleep, and 10 points represented the baryodynia

### 2.8. Statistical Treatment

In this study, the experimental data were processed by SPSS 20.0, and GraphPad Prism 7 (GraphPad software, San Diego, USA) was used to draw pictures of the data. The enumeration data and measurement data were tested by *x*^2^ and *t*-test. When *p* < 0.05, the differences were considered to be statistically significant.

## 3. Results

### 3.1. Comparison of Patients' General Information

There was no significant difference in the general information between the two groups, see details in Table 1.

### 3.2. Comparison of Patients' BMD Values

The BMD values of the lumbar vertebrae L_2-4_, total hip, and femur neck at 6 months and 1 year after treatment in the experimental group were significantly higher than those in the control group (*p* < 0.001), see details in Figure 1.

### 3.3. Comparison of Patients' Pain Indexes

There was no statistical difference in the pain scores between the experimental group and the control group before treatment (7.65 ± 0.64 vs. 7.65 ± 0.55, *p* > 0.05). The pain scores at 6 months and 1 year after treatment in the experimental group were significantly lower than those in the control group (4.24 ± 0.55 vs. 5.67 ± 0.61, 3.01 ± 0.44 vs. 4.13 ± 0.62, *p* < 0.001).

## 4. Discussion

Due to the existence of degenerative deformation during the senescence of the body, the calcium absorption rate in gastrointestinal tract and the sex hormone levels will decrease with age [13], so that age is a risk factor for osteoporosis, and higher age is associated with a higher incidence of osteoporosis [14]. Epidemiological data have shown that the number of elderly patients with osteoporosis is close to 100 million ranking third in chronic diseases among residents, and the incidence of osteoporotic fractures is as high as 7.5% in China. The rate of hip fracture in elderly patients increased by three times during 2012-2016, and the mortality of patients within one year is as high as 20.0%. In addition, this number will continue to rise further with the aggravation of the population aging in China [15–17]. Early measures of prevention and treatment can effectively improve the quality of life in elderly patients with osteoporosis and reduce the medical burden in China. At present, the calcium treatment is the basic treatment for senile osteoporosis. Calcium, as a key component of bone, plays an important role in reducing the osteoporosis. Some studies have shown that calcium can prevent the age-related calcium deficiency, thereby exerting the effect on prevention and treatment of senile osteoporosis [18]. However, the effect of calcium alone is limited, and it is necessary to cooperate with other therapeutic agents. At present, the common therapeutic agents used for osteoporosis also include bisphosphonates, calcium, and sex hormone supplementation. Bisphosphonates can maintain the effect on antiosteoporotic fracture for several years even after discontinuation, while the antifracture efficacy of other drugs decreases, indicating that bisphosphonates have a favorable value in long-term antiosteoporosis [19].

Scholars Tim et al. have found that the treatment with bisphosphonates for 4 years can reduce the risk of hip fracture by 50.0%. The annual growth rate of BMD value is 1.0% at a daily dose of 150 mg, and the densities of lumbar vertebrae and hip can increase continuously [20]. The results of this study showed that the densities of lumbar vertebrae, total hip, and femur neck in the two groups were increased after the treatment of bisphosphonates and calcium. However, the BMD values of lumbar vertebrae L_2-4_, total hip, and femur neck in the experimental group at 6 months and 1 year after treatment were significantly higher than those in the control group (*p* < 0.001), suggesting that the intensity of pamidronate disodium by intravenous injection was higher than that of alendronate sodium by oral administration. Pamidronate disodium can fully adhere to the surface of trabecular bone by intravenous injection, which can directly inhibit the phagocytic factors of osteoclasts, hinder the effects of osteoclasts on dissolution and destruction of bone, and slow down the bone absorption, thereby preventing the bone dissolution [21]. Baroncelli et al. have believed that pamidronate disodium can promote the bone formation in patients with spontaneous juvenile osteoporosis, improve the BMD, reduce the incidence of fractures, and prevent the disability after fractures [22]. In addition, pamidronate disodium has the analgesic effect, especially in relieving the symptoms of bone pain. It can inhibit the premature maturation of osteoclasts, slow down the release frequencies of nociceptive transmitters such as prostaglandins and lactic acid and inflammatory transmitters, and relieve the osteolytic pain [23]. At present, pamidronate disodium is often used for analgesia in bone metastasis of malignant tumor. Some scholars have believed that the analgesic effect of this drug in osteoporosis is better than that in bone metastasis of malignant tumor [24]. This study showed that the pain scores at 6 months and 1 year after treatment in the experimental group were significantly lower than those in the control group (*p* < 0.001), indicating that pamidronate disodium has a definite analgesic effect in elderly patients with osteoporosis, which can effectively reduce the patients' severity of pain and has a great significance for improving the quality of life.

It is worth noting that the elderly patients with chronic diseases have the characteristic of poor medical compliance behavior [25], and patients with osteoporosis need long-term medication. In clinic, it is generally agreed that the treatment time of osteoporosis should be more than 1 year. Therefore, no matter what kind of drugs are used, attention should be paid to maintain the medication compliance of patients to ensure that drugs can play the best effect. Based on the mobile terminal platform for the Internet of Things, this study established a remote monitoring platform for elderly patients with osteoporosis and realized the continuous management of elderly patients, so that the medication effects of the two groups were better. With the development of aging society, the importance of information construction in elderly chronic diseases is increasingly prominent. It is beneficial for elderly patients with osteoporosis to accelerate the construction of the mobile terminal platform for the Internet of Things, and elderly patients with chronic diseases also benefit more.

In conclusion, the treatment of pamidronate disodium combined with calcium based on the mobile terminal platform for the Internet of Things can reduce the severity of pain in elderly patients with osteoporosis and improve the BMD, which has a generalization value.

## Figures and Tables

**Figure 1:** Comparison of patients' BMD values (^−^*x* ± *s*, g/cm^2^). Notes were as follows: Figure 1(a) shows the BMD value of L_2_.  Figure 1(b) shows the BMD value of L_3_.  Figure 1(c) shows the BMD value of L_4_.  Figure 1(d) shows the BMD value of total hip.  Figure 1(e) shows the BMD value of femur neck. There was no statistical difference in the BMD values of lumbar vertebrae L_2-4_, total hip, and femur neck between the experimental group and the control group before treatment (0.74 ± 0.05 vs. 0.75 ± 0.05, 0.75 ± 0.04 vs. 0.74 ± 0.04, 0.77 ± 0.05 vs. 0.78 ± 0.04, 0.62 ± 0.05 vs. 0.63 ± 0.05, 0.58 ± 0.04 vs. 0.59 ± 0.03, *p* > 0.05). The BMD values of lumbar vertebrae L_2-4_, total hip, and femur neck in the experimental group at 6 months after treatment were significantly higher than those in the control group (0.84 ± 0.03 vs. 0.77 ± 0.04, 0.83 ± 0.04 vs. 0.78 ± 0.03, 0.90 ± 0.04 vs. 0.84 ± 0.06, 0.69 ± 0.04 vs. 0.64 ± 0.03, 0.68 ± 0.03 vs. 0.62 ± 0.04, *p* < 0.001). The BMD values of lumbar vertebrae L_2-4_, total hip, and femur neck in the experimental group at 1 year after treatment were significantly higher than those in the control group (0.95 ± 0.02 vs. 0.82 ± 0.03, 0.96 ± 0.05 vs. 0.81 ± 0.06, 1.04 ± 0.08 vs. 0.86 ± 0.04, 0.71 ± 0.03 vs. 0.65 ± 0.04, 0.70 ± 0.03 vs. 0.63 ± 0.04, *p* < 0.001).

**Table 1:** Comparison of patients' general information.

Groups	Experimental group (*n* = 68)	Control group (*n* = 52)	*X* ^2^/*t*	*p*
Gender			0.175	0.676
Male	34	28		
Female	34	24		
Age (years)	73.99 ± 3.16	74.44 ± 3.65	0.723	0.471
Body mass (kg)	62.65 ± 2.65	62.74 ± 2.40	0.192	0.848
BMI (kg/m^2^)	22.11 ± 1.20	22.13 ± 1.24	0.089	0.929
Course of disease (years)	5.29 ± 1.94	4.98 ± 1.66	0.922	0.358
Severity degree			0.369	0.544
Moderate grade	48	34		
Severe grade	20	18		
Education level				
Primary school	30	26	0.410	0.522
Senior high school	28	20	0.091	0.764
University and above	10	6	0.256	0.613
Income level (yuan)			0.019	0.890
≥4000	41	32		
<4000	27	20		
Payment of medical expenses				
Medical insurance	30	22	0.039	0.843
Commercial insurance	24	18	0.006	0.938
Others	14	12	0.108	0.743
Place of residence			0.016	0.901
Town	40	30		
Countryside	28	22		

## Data Availability

Data to support the findings of this study is available on reasonable request from the corresponding author.
